# Chronic Treatment with Atrial Natriuretic Peptide in Spontaneously Hypertensive Rats: Beneficial Renal Effects and Sex Differences

**DOI:** 10.1371/journal.pone.0120362

**Published:** 2015-03-16

**Authors:** Mariana Romero, Carolina Caniffi, Gonzalo Bouchet, María A. Costa, Rosana Elesgaray, Cristina Arranz, Analía L. Tomat

**Affiliations:** Cátedra de Fisiología, Facultad de Farmacia y Bioquímica, Universidad de Buenos Aires, IQUIMEFA-CONICET, Junín 956, piso 7, 1113 Ciudad de Buenos Aires, Argentina; University of Southampton, UNITED KINGDOM

## Abstract

**Objective:**

The aim of this study was to investigate the effects of chronic treatment with atrial natriuretic peptide (ANP) on renal function, nitric oxide (NO) system, oxidative stress, collagen content and apoptosis in kidneys of spontaneously hypertensive rats (SHR), as well as sex-related differences in the response to the treatment.

**Methods:**

10 week-old male and female SHR were infused with ANP (100 ng/h/rat) or saline (NaCl 0.9%) for 14 days (subcutaneous osmotic pumps). Systolic blood pressure (SBP) was recorded and diuresis and natriuresis were determined. After treatment, renal NO synthase (NOS) activity and eNOS expression were evaluated. Thiobarbituric acid-reactive substances (TBARS), glutathione concentration and glutathione peroxidase (GPx) and superoxide dismutase (SOD) activities were determined in the kidney. Collagen was identified in renal slices by Sirius red staining and apoptosis by Tunel assay.

**Results:**

Female SHR showed lower SBP, oxidative stress, collagen content and apoptosis in kidney, and higher renal NOS activity and eNOS protein content, than males. ANP lowered SBP, increased diuresis, natriuresis, renal NOS activity and eNOS expression in both sexes. Renal response to ANP was more marked in females than in males. In kidney, ANP reduced TBARS, renal collagen content and apoptosis, and increased glutathione concentration and activity of GPx and SOD enzymes in both sexes.

**Conclusions:**

Female SHR exhibited less organ damage than males. Chronic ANP treatment would ameliorate hypertension and end-organ damage in the kidney by reducing oxidative stress, increasing NO-system activity, and diminishing collagen content and apoptosis, in both sexes.

## Introduction

It is well established that blood pressure is higher in men than age-match premenopausal women. However, after menopause, the prevalence of hypertension in women is higher than it is in men [1, 2]. Moreover, progression of hypertensive renal disease tends to be milder in females, with a favorable influence in the physiopathology of hypertension and secondary kidney damage [3, 4].

Atrial natriuretic peptide (ANP) is mainly expressed and stored in granules in the heart atria and elicits its effects by binding primarily with A-type natriuretic peptide receptor (NPR-A) and inducing natriuresis, diuresis and vasorelaxation, [5, 6]. The actions of this peptide involve an increase in glomerular filtration rate, inhibition of sodium and water reabsorption, and a reduction in renin secretion [6]. Nishikimi T et al. have demonstrated, in mice, that ANP has antifibrotic effects on the kidney, involving the activation of NPR-A and/or C-type natriuretic peptide receptor (NPR-C), producing an increase in renal cGMP levels and a decrease in transforming growth factor beta (TGF-β) expression and collagen I and III content [7]. Further, in our laboratory we provided evidence that ANP exerts a hypotensive effect through enhancement of cardiovascular and renal NOS activity, in both, normotensive and hypertensive rats [8–10].

Little is known about the relationship between natriuretic peptides and reactive oxygen species (ROS) in renal physiopathology. It has been reported that ANP counteracts ROS generation in aortic smooth muscle cells and inhibits ROS-induced cell damage via the GC-A/cGMP pathway [11, 12]. Renal oxidative stress can be a cause, a consequence, or more likely a potentiating factor for hypertension. While animal and human studies have established that ANP reduces oxidative stress in the cardiovascular system, in hypertension its antioxidant effect on the kidney has not been established yet [13–15].

Depending on the experimental conditions and cell context, ANP has antiapoptotic or proapoptotic properties [16]. In a recent study we have described that chronic treatment with ANP promotes antiapoptotic effects on the heart in SHR of both sexes, and this is accompanied by a reduction in cardiac oxidative stress, fibrosis and hypertrophy [14].

Different authors have shown that estrogens exhibit antioxidant, antiapoptotic and antiproliferative effects and that these actions are mediated, in part, by NO-system activation [17–19]. These sexual hormones protect against the development of glomerulosclerosis in a model of subtotal renal ablation in female rats [20]. In addition, estradiol decreases the local synthesis of angiotensin-II, endothelin-1, free radicals and lipid peroxides in the kidney [21].

Taking into account this background and our previous studies showing that ANP has cardiac benefits in hypertensive animals [14], we hypothesized that long-term treatment with ANP induces renal benefits in SHR and that there are sex differences in the response to this chronic treatment. Therefore, we proposed to investigate morphological changes as well as, antioxidant and antiapoptotic effects of chronic treatment with ANP on the kidney of SHR rats, and whether sex differences existed.

## Materials and Methods

### Animals

Ten-week-old male and female SHR were purchased from Instituto de Investigaciones Médicas A. Lanari, Facultad de Medicina (Universidad de Buenos Aires, Argentina). Rats were housed in a humidity and temperature-controlled environment with an automatic 12-hour light-dark cycle. They were fed standard rat chow from Nutrimentos Purina (Buenos Aires, Argentina) and tap water ad libitum up to the day of the experiments.

### Experimental design

All experimental protocols were performed in accordance with the Guide for the Care and Use of laboratory Animals (National Institutes of Health, Publication No. 85-23, Revised 1996) and with regulation 6344/96 of Argentina‘s National Drug, Food and Medical Technology Administration (ANMAT). Experimental procedures were approved by the Ethics Committee of the School of Biochemistry and Pharmacy (CEFFB), Universidad de Buenos Aires, Buenos Aires, Argentina.

### Protocol

Animals were separated by sex and then randomly assigned to the ANP treated group (n = 12): chronic infusion with ANP (100 ng/h/rat), or the Control group (n = 12): chronic infusion with NaCl 0,9%, during 14 days. Chronic infusion in both groups was performed using Alzet micro-osmotic pumps (Model 1002), prepared according to the manufacturer’s instructions and implanted subcutaneously between the scapulae using aseptic technique under light ether anaesthesia.

Systolic blood pressure (SBP) was recorded, 24-hour urine volume was measured and urine samples were collected at the end of the experimental period in all groups of animals. SBP was measured in awake animals (tail cuff method) with a MP100 Pulse Transducer, PanLab (Quad Bridge Amp, ADInstruments), and recorded with a polygraph (Quad Bridge Amp, ADInstruments). Data were obtained using data acquisition software (PowerLab 8/30 and Labchart, Australia).

Animals were placed in metabolic cages for adaptation to the environment two days before the beginning of the experiment; after the adaptation period animals were weighed and placed in metabolic cages in order to collect 24-hour urine. Diuresis was determined gravimetrically and urinary sodium concentration was measured with an ion analyser (Tecnolab, Model T-412). The concentration of nitrites and nitrates (NOx), end products derived from NO metabolism, was determined according to the procedure described by Verdon et al. [22].

Animals were, subsequently euthanized by decapitation and the kidneys were removed and weighed, in order to evaluate NOS activity and expression, oxidative stress, collagen content and apoptosis.

### Determination of NOS activity

Tissue NOS activity was measured using [^14^C] L-arginine as substrate, as described previously [23, 24]. 2–3 mm thick tissue slices were incubated in Krebs solution with 0.5 μCi/ml [^14^C] L-arginine for 30 minutes at 37°C. The reaction was stopped by adding 500 μl stop buffer containing 0.5 mM EGTA, 0.5 mM EDTA and 20 mM HEPES (pH 5.5). Tissue samples were then homogenized in the stop solution and the homogenates were centrifuged at 12,000 g for 20 minutes.

The supernatants were then applied to a 1ml Dowex AG 50W-X8 column (Na^+^ form, Bio-Rad), hydrated with the stop buffer, and eluted with 2 ml of distilled water. The amount of [^14^C] L-citrulline was determined with a liquid scintillation counter (Wallac 1414 WinSpectral). Specific NOS activity was assessed in the presence of 10^−4^ M L-NAME (Sigma). NO production in each tube was normalized to the weight of the tissue slices incubated with the substrate during equal periods of time and expressed as picomoles of [^14^C] L-citrulline per gram wet weight per minute.

### Western blot analysis

Samples of medulla and cortex from kidney tissue containing equal amounts of protein (0.10 mg protein/lane) were separated by electrophoresis in 7.5% SDS-polyacrylamide gels, transferred to a nitrocellulose membrane (Bio-Rad, Munich, Germany), and then incubated with rabbit polyclonal anti-eNOS antibodies (1/500 dilution, epitope at the NH_2_ terminus, Santa Cruz Biotechnology, Santa Cruz, CA) and a horseradish peroxidase-conjugated goat anti-rabbit secondary antibody (1/5,000 dilution BioRad Laboratories, USA). A marker of β-actin was used as a loading control and data were normalized to β-actin expression. Samples were revealed by chemiluminescence using an enhanced chemiluminescence reagent (Amersham Pharmacia Biotechnology, Uppsala, Sweden) for 2–4 minutes. A quantification of the bands was performed by digital image analysis using a Hewlett-Packard scanner and Totallab analyzer software (Biodynamics, Seattle, WA). All experiments were performed in triplicate [14].

### Oxidative stress evaluation

Slices from cortex and medulla of the kidneys were homogenized (OMNI MIXER homogenizer) in 30 mM phosphate buffer potassium, pH 7.4, 120 mM KCl (1g tissue/10 ml buffer). Lipid oxidative damage was assessed by measuring the extent of formation of 2-thiobarbituric acid reactive substances (TBARS) [25]. Super oxide dismutase (SOD) activity was assessed by measuring the ability of the homogenate to inhibit autoxidation of epinephrine and was expressed as units of SOD per milligram of protein [26]. Catalase (CAT) activity was determined by the conversion of hydrogen peroxide to oxygen and water and was expressed as picomoles per milligram of protein [27]. The assay described by Flohé and Gunzler was used to measure glutathione peroxidase (GPX) activity and it was expressed as nanomoles per minute per milligram of protein [28].

In order to measure glutathione content, tissue slices were homogenized in 100 mM phosphate buffer sodium, pH 7.0, 5 mM EDTA (1.6 g tissue/10 ml buffer), and centrifuged at 13.000 rpm for 20 minutes at 4°C. Glutathione concentration was measured according to the method described by Tietze F. and was expressed as milligram per milligram of protein [29]. Protein concentration was determined by the method of Bradford et al. [30].

### Histological evaluation and Tunel Assay

Kidneys were cut longitudinally, fixed in phosphate-buffered 10% formaldehyde, pH 7.2, and embedded in paraffin wax.Kidney sections (3μm) were subjected to collagen-specific Picrosirius Red staining as described previously [31]. Collagen staining was evaluated following a score: 0 = normal and slight staining surrounding tubular, glomerular and vascular structures; 1 (mild) = weak staining, that doubles normal label, surrounding tubular, glomerular, and vascular structures; 2 (moderate) = moderate staining in the peritubular interstitium and inside glomeruli; 3 (severe) = strong staining that replaces glomerular and tubular structures, compromising <25% of the cortical area; and 4 (very severe) = strong staining that replaces glomerular and tubular structures, compromising >25% of the cortical area. A score was assigned to each section, mainly reflecting the changes in extent rather than intensity of staining.

The DeadEnd Colorimetric TUNEL System, a nonradioactive kit designed to end-label fragmented DNA of apoptotic cells, was used as previously described [32]. The number of TUNEL-positive cells was counted in 20 visual fields (magnification X400) for each rat.

Histological and TUNEL assays were analyzed using an Olympus BX51 light microscope equipped with a digital camera (QColor 3, Olympus America, Inc., Richmond Hill, Ontario, Canada) connected to the Image-Pro Plus 4.5.1.29 software (Media Cybernetics, LP, Silver Spring, MD, USA). Measurements were performed blindly and under similar light, gain, offset, and magnification conditions.

### Statistical Analysis

All values are expressed as means ± SEM. The Prism program (Graph Pad Software, Inc., San Diego, CA, USA) was used for statistical analysis. The mean and standard error of median values of each variable were calculated for each group. The results of each variable for each experimental group were analysed with a two-way analysis of variance (ANOVA) where one factor was the different treatments and the other was sex (male or female). The effects of one factor were tested independently of the effects of the other, as well as the interaction between both factors. No interaction between treatments and genotype was found. Multiple comparisons were performed using a Bonferroni post hoc test. p value < 0.01 was considered a significant difference.

## Results

### Effect of chronic treatment with ANP on SBP, diuresis, natriuresis and NO system

According to our previous findings, SBP was higher in male than in female rats, and chronic treatment with ANP reduced this parameter in both sexes (Table 1). We found no differences between sexes in diuresis and natriuresis between sexes, although ANP treatment increased both parameters in male and female rats (Table 1). Renal response to ANP treatment was more marked in female than in male SHR (increase in urine volume: Male: 76% and female: 87%; increase in urinary sodium Male: 87% and female: 139%). ANP treatment induced no changes in kidney weight in either male or female rats. We evaluated NOx excretion as an indicator of NO systemic production. We observed that female SHR presented higher NOx excretion in 24-hour urine than male rats, with increased NOx excretion in both sexes after treatment with ANP (NOx (nmol/min.100g): Control male: 2.6 ± 0.2, Control female: 3.4 ± 0.3*, ANP male: 3.8 ± 0.6*, ANP female: 4.5 ± 0.4†; *p<0.01 vs Control male; †p<0.01 vs Control female).

**Table 1:** Effect of chronic treatment with ANP on blood pressure, kidney weight, diuresis and natriuresis in SHR of both sexes.

	Male		Female	
	Control	ANP	Control	ANP
**BW (g)**	303±6	295±8	210±4*	209±4
**KW/BW (g/g)**	0.42±0.05	0.43±0.04	0.41±0.02	0.41±0.03
**SBP (mmHg)**	209±8	191±7*	181±6*	168±6^†^
**UV (ml/100g.24h)**	3.4±0.5	6.0±0.7*	3.9±0.7	7.3±0.5^†^ ^‡^
**U_Na_V (mEq/24hs)**	0.96±0.10	1.80±0.13*	0.93±0.11	2.22±0.15^†^ ^‡^

BW: body weight; KW: kidney weight; SBP: systolic blood pressure; UV: urinary volume; U_Na_ V: urinary sodium.

Value represents mean ± SEM (n = 12).

*p < 0.01 vs Control Male

^†^p<0.01 vs Control Female

^‡^p<0.01 vs ANP male

In order to verify whether the increase in NOx was due to an increase in activity and/or expression of NOS, NOS activity and expression in renal medulla and cortex was studied to determine existence of sex differences Fig. 1. Renal activity of the enzyme was higher in female than in male SHR. Chronic treatment with ANP increased NOS activity in renal medulla and cortex in both sexes Fig. 1A. The increase of renal NOS activity in response to ANP treatment was more marked in female than in male SHR (Changes in NOS activity induced by ANP treatment (pmol/min.100g): Renal cortex: Male: 90.5±10.2 vs Female: 180.4±15.9*; Renal medulla: Male: 89.3±8.5 vs Female: 155.7±12.2*; *p< 0.01). Kidney eNOS protein content was higher in female than in male SHR, and ANP increased eNOS expression in both sexes Fig. 1B and C.

**Fig 1:** Effects of ANP treatment on renal NOS. (A) Nitric oxide synthase (NOS) activity; (B) Representative blots of eNOS and β-actin; (C) Quantification of eNOS bands. All experiments were performed in triplicate. β-actin was used as a loading control and data are normalized to actin expression. White spaces demarcate noncontiguous gel lanes. Data are mean ± SEM (n = 12). *p<0.01 vs Control male, ^†^p<0.01 vs Control female.

### Study of renal oxidative stress in response to chronic treatment with ANP

Female kidneys showed less oxidative stress than male ones and displayed higher levels of glutathione and lower content of TBARS when compared to the male group Fig. 2A and B. Chronic treatment with ANP increased the levels of glutathione and reduced TBARS in kidneys of both sexes. The study of antioxidant enzymes showed that renal activity of CAT was higher in female than male rats. Renal GPx and SOD activities in female rats were lower when compared to the male group. Chronic treatment with ANP increased GPx and SOD activities in both sexes (Table 2).

**Fig 2:** Effects of ANP treatment on renal concentration of glutathione and TBARS. (A) Glut: glutathione; (B) TBARS: thiobarbituric acid reactive substances. Data are mean ± SEM (n = 12). *p <0.01 vs Control male, ^†^p<0.01 vs Control female.

**Table 2:** Effect of chronic treatment with ANP on the enzymes involved in renal oxidative state of male and female SHR.

	Male		Female	
	Control	ANP	Control	ANP
**CAT (pmol/mg.prot)**	0.85±0.06	0.99±0.08	1.33±0.12*	1.41±0.11
**SOD (USOD/mg.prot)**	8.1±0.6	10.1±0.5*	6.2±0.4*	8.6±0.6†
**GPx(μmol/min.mg.prot)**	210±21	307±37*	81±9*	157±15†

CAT: Catalase; SOD: superoxide dismutase; GPx: glutathione peroxidase.

Value represents mean ± SEM (n = 12).

*p <0.01 vs control male

†p<0.01 vs control female

### Sirius Red staining and apoptosis in kidney

Male renal cortex and medulla showed a greater staining for collagen, compared to female rats. Treatment with ANP reduced collagen content in both tissues and sexes Fig. 3A and B. Examination of TUNEL-stained kidney sections revealed fewer apoptotic cells in cortex and medulla of female rats compared to males. ANP treatment decreased the number of apoptotic cells in renal cortex and medulla in both sexes Fig. 3E and F.

**Fig 3:** Sirius Red staining and TUNEL positive apoptotic nuclei in kidney after treatment with ANP. (A) The red colour of Sirius red staining under the light microscope indicates total collagen deposits, representative images are from renal cortex of each group; (B) Sirius red Score values; (C) Representative micrographs of TUNEL staining in renal cortex and medulla; (D) Apoptotic cells quantification. C-M: Control male; ANP-M: ANP male; C-F: Control female; ANP-F: ANP female. All images are at the same magnification (400X). Scale bar: 30 μm. Value represents mean ± SEM (n = 12) *p <0.01 vs Control male, ^†^p<0.01 vs Control female.

## Discussion

In the present study we demonstrated that chronic treatment with ANP exerts beneficial effects in kidney of SHR, reducing oxidative stress, collagen content and apoptosis. These actions were also accompanied by an increase in renal NO-system activity. Moreover, we found that important sex differences exist in this model of hypertension and in the response to chronic ANP treatment.

It is well known that ANP modulates arterial blood pressure through different mechanisms that involve the control of sodium and water excretion, in addition to vasorelaxation. As expected, chronic treatment with ANP decreased SBP and increased sodium and water excretion. In previous studies we found that these actions of ANP involved, at least in part, an increase in renal NOS activity by interacting with natriuretic receptors NPR-A and NPR-C in both normotensive and hypertensive male animals [33].

Our results showed no differences between sexes in diuresis and natriuresis of control groups. However, the effects of ANP in these parameters were more marked in females. In this regard, Reckelhoff et al. reported that male SHR not only have higher SBP but also a blunted pressure-natriuresis relationship compared with female SHR [34]. Although the mechanism responsible for the sexual dimorphism in renal function is unknown, this fact could be attributed to the beneficial effects of estradiol on kidney function, which include higher eNOS activity in renal vasculature and tubular cells and a reduction in oxidative stress [35–38].

Adding to this, chronic ANP increased the activity of renal NOS and eNOS expression in male and female SHR rats. However, the response of renal NOS to ANP in female rats was higher than in males, indicating that the presence of estrogens could improve the effect of ANP on NO-system. Moreover, control female SHR showed not only higher NOx levels, as report previously [14], but also an increase in the activity and expression of eNOS in renal cortex and medulla, as well as reduction in kidney oxidative stress compared to male rats, indicating a sex difference in these parameters.

Experimental and human hypertensive studies documented that NO deficiency mediates oxidative stress in the kidney [39–41]. Moreover, it was reported that oxidative stress and renal NO deficiency contributes to the hypertensive state in SHR [42, 43]. Adding to this, previous studies showed that hypertension is ameliorated or reverted in this model after use of an oxygen radical scavenger [44, 45].

Furthermore, it has been shown, both in humans and animals, that NO level is higher in females because estrogens not only stimulate NO production but also decrease inactivation of NO by oxygen radicals [35, 46, 37]. Moreover, epidemiological and experimental evidence suggests that oxidative stress is enhanced in males compared with females [47, 48]. Additionally, estradiol protects the female kidney in part by attenuating injury-induced increases in renal superoxide production [49]. Our results show that kidney of female SHR exhibits higher levels of glutathione and lower content of TBARS than male ones, indicating a sex difference in renal oxidative status. The increased production of renal free radicals could explain the higher lipid peroxidation and the lower levels of glutathione content observed in males. Consequently, we observed increased activity of antioxidant enzymes, SOD and GPx in male kidneys of SHR as a compensatory response. In this regard, the increased levels of superoxide anion and H_2_O_2_ would enhance SOD and GPx activities, respectively. These results are consistent with previous reports by Sullivan et al. showing that male SHR exhibit greater SOD activity and higher H_2_O_2_ levels in renal inner medulla than females [50, 5].

Although, the antioxidant role of ANP has been established in cardiovascular, liver and immune system diseases, little is known about the relationship between ANP and oxidative stress in renal injury [13]. Ogawa Y et al. recently observed that the administration of aldosterone in NPR-A-deficient mice caused a mayor increase in hypertension, glomerular injury and ROS than in wild type mice, suggesting a protective role of ANP [51]. In our study, we found that chronic treatment with ANP decreased oxidative stress in kidney of SHR, reducing lipid peroxidation in males and increasing glutathione levels in both sexes. Furthermore, these effects are due to the increase in GPx and SOD activities induced by the peptide in both sexes.

In the present study, we also demonstrated that chronic treatment with ANP decreased the deposit of collagen in medulla and cortex in both sexes. The increase of NO production as well as the decrease in renal oxidative stress observed in these animals could explain, at least in part, these renal effects of ANP. According to our results, it has been recently found that mice carrying a target disruption of a gene coding for NPR-A receptor exhibit renal fibrosis and remodeling, accompanied by an increase in the expression of TGF-β [52].

Moreover, kidneys of females showed minor staining for collagen in both medulla and cortex compared to males. Once more, this could be explained by the fact that estrogens are known to be nephroprotective not only by decreasing oxidative stress but also by reducing the generation and deposit of extracellular matrix protein, and by diminishing the expression of TGF-β [20].

Ortiz et al. have reported that apoptosis of the intrinsic renal cells plays an important role in the persistence and progression of renal injury [53]. In this regard, the present protocol represents the first in vivo study that analyzes the effects of ANP treatment on apoptosis in the kidney, showing that chronic treatment with the peptide reduces apoptosis in renal medulla and cortex of both male and female SHR. In previous studies, we demonstrated that ANP treatment reduces apoptosis in the cardiac ventricle of both male and female SHR [14].

On the other hand, our results showed that females exhibited less apoptosis in renal medulla and cortex than males. These results are probably due to the fact that estradiol regulates different components of the apoptotic pathway by modulating their expression or activity in diverse tissues and experimental models [54, 55]. Although, we recently observed that there were no differences between males and females in the number of apoptotic cells in left ventricle [14], our present results in kidney are the first evidence of a sex difference in apoptosis in SHR.

## Conclusions

In summary, we have demonstrated that the kidney of female SHR presents less collagen deposit, apoptosis and oxidative stress in this model of hypertension. Taking into account that NO exerts antioxidant and antifibrotic effects [56, 57], along with our previous findings linking ANP and eNOS activation, we can postulate that indirect effects of ANP in kidney would be mediated, at least in part, by the increase in NO, which also contributes to reduce oxidative stress.

Whether sex plays an essential role in the onset of hypertension complications and organ damage continues to be an issue of intense debate, but we found that, in this model of hypertension, female SHR showed less signs of early fibrosis, apoptosis and oxidative stress in the kidney than male SHR. While we must take into account that males exhibit higher blood pressure values than females, it is important to consider that blood pressure values in females are also consistent with target organ damage. On the other hand, chronic treatment with ANP not only lowered SBP but also induced antifibrotic, antiproliferative and antiapoptotic effects in the kidney of male and female SHR. In accordance with our results, the beneficial effects of ANP in hypertension probably involve activation of the NO-system and an improvement in the antioxidant system.
